This article has been retracted.

# Effect of Tumor Microenvironment and Angiogenesis on Clinical Outcomes of Primary Central Nervous System Lymphoma

**DOI:** 10.1155/2021/3291762

**Published:** 2021-09-30

**Authors:** Hui-Ching Wang, Hui-Hua Hsiao, Jeng-Shiun Du, Shih-Feng Cho, Tsung-Jang Yeh, Yuh-Ching Gau, Yi-Chang Liu, Sin-Hua Moi

**Affiliations:** ^1^Graduate Institute of Clinical Medicine, College of Medicine, Kaohsiung Medical University, Kaohsiung 807, Taiwan; ^2^Division of Hematology and Oncology, Department of Internal Medicine, Kaohsiung Medical University Hospital, Kaohsiung Medical University, Kaohsiung 807, Taiwan; ^3^Faculty of Medicine, College of Medicine, Kaohsiung Medical University, Kaohsiung 807, Taiwan; ^4^Center of Cancer Program Development, E-Da Cancer Hospital, I-Shou University, Kaohsiung 824, Taiwan

## Abstract

Primary central nervous system lymphoma (PCNSL) is a rare lymphoma, and the disease course is often aggressive with poor prognosis outcomes. PCNSL undergoes germinal center reactions and impairs B-cell maturation. However, angiogenesis is also involved in the tumorigenesis and progression of PCNSL. This study investigated the effects of the tumor microenvironment and angiogenesis-associated genomic alterations on the outcomes of PCNSL. The analysis also evaluated the influence of treatment modality and timing on PCNSL survival using partial least squares variance-based path modeling (PLS-PM). PLS-PM can be used to evaluate the complex relationship between prognostic variables and disease outcomes with a small sample of measurements and structural models. A total of 19 immunocompetent PCNSL samples were analyzed by exome sequencing. Our results suggest that the timing of radiotherapy and mutations of *ROBO1* and *KAT2B* are potential indicators of PCNSL outcomes and may be affected by baseline characteristics such as age and sex. Our results also showed that patients with no mutations of ROBO1 and KAT2B, SubRT subgroup showed favorable survival outcomes compared with no SubRT subgroup in short-term follow-up. All SubRT patients have received high-dose methotrexate induction chemotherapy in the initial treatment. Therefore, initial induction chemotherapy combined with subsequent radiotherapy might improve survival outcomes in PCNSL patients who have no ROBO1 and KAT2B somatic mutations in short-term follow-up. The overall findings suggest that the tumor microenvironment and angiogenesis-associated genomic alterations and treatment modalities are potential indicators of overall survival and may be affected by the baseline characteristics of PCNSL patients.

## 1. Introduction

Primary central nervous system lymphoma (PCNSL) is a rare brain tumor characterized by extranodal non-Hodgkin's lymphoma (NHL), which arises from the CNS with lymphoma cells localized in the perivascular areas. The major histology of PCNSL is diffuse large B-cell lymphoma [1], and PCNSL accounts for less than 1% of non-Hodgkin lymphomas [2]. The histogenetic origin of PCNSL indicates their involvement in germinal center reactions and that further B-cell maturation is impaired, which corresponds to activation of somatic hypermutation (SHM) in B-cell receptor (BCR) heavy and light chains [3].

The standard treatment for diffuse large B-cell lymphoma is ineffective in PCNSL, including the R-CHOP regimen. Whole-brain radiotherapy (WBRT) demonstrates its efficacy in PCNSL patients, but disease recurrence and neurotoxicity occur significantly during the follow-up period [4]. High-dose induction chemotherapy with methotrexate (HD-MTX) serves as a cornerstone of treatment for PCNSL and achieves long-term survival benefits [5]. Subsequential WBRT combined with stem cell transplantation has been regarded as a consolidation therapy; however, subsequential WBRT might have a negative impact on cognitive function [6, 7]. Targeted therapy based on the molecular mechanisms that trigger PCNSL has been developed in recent years. The role of rituximab, a monoclonal antibody targeting CD20, in PCNSL is still debated, with divergent views expressed on both sides of the efficacy [8–10]. Some other pathways, including Bruton's tyrosine kinase (BTK), BCR/Toll-like receptor, and phosphoinositide 3-kinase (PI3K)/mechanistic target of rapamycin (mTOR) signaling, are under investigation and research [2–4].

Angiogenesis plays an important role in tumorigenesis in various types of malignancies. Vascular endothelial growth factor (VEGF) is associated with the prognosis and management of NHL [11]. Higher expression of VEGF was correlated with poor prognosis and treatment response in lymphoma patients, which implies vessel formation. Hormones associated with blood vessels are tightly connected with NHL [12]. Together with angiogenic factors, other tumor microenvironment components, such as immune cells, endothelial progenitor cells, and stromal cells, are pivotal in the tumorigenesis and progression of lymphoproliferative disorders [13]. In both high-grade and low-grade NHL, tumors develop transluminal bridges, exhibit intussusceptive microvascular growth, and distinguish the mode of tumor vessel growth [14]. These results suggest that angiogenesis and the vascular-associated microenvironment may be tightly involved in PCNSL.

The partial least squares (PLS) approach is a commonly used method in chemical modeling that considers the optimal number of latent variables (nLVs) [15]. The PLS path model, which consists of construct measurement and structural relationships, can integrate categorical variables. However, overfitting is the most important problem in PLS path modeling (PLS-PM); appropriate variable selection can lower the risk of overfitting by reducing the dimensionality of the variable space [5, 6]. The PLS-PM results are useful for exploratory and confirmatory research. PLS-PM is more flexible in dealing with small sample sizes and examining latent variables [7]. The angiogenesis-related genes involved in the estimation of overall survival can be associated with various latent variables according to the characteristics, including baseline characteristics and treatment modalities. Therefore, the influence of different latent variables on survival status can be measured using the PLS-PM measurement and structural models.

Studies have reported an association between angiogenesis and prognosis in PCNSL [16, 17]. However, the effects of baseline characteristics, genomic profiles, and treatment modalities on overall survival and outcomes of PCNSL have not been studied. In our study, we aimed to use a PLS variance-based path modeling approach to investigate the influence of baseline characteristics, genomic profiles, and treatment modalities thoroughly and comprehensively on survival outcomes in PCNSL.

## 2. Materials and Methods

### 2.1. Data Sets

This is a retrospective study. A total of 19 immunocompetent PCNSL samples with exome sequencing (WES) were included [18]. One patient was excluded due to a lack of clinical characteristics, so 18 patients were analyzed. The clinical characteristics, including diagnosis age, sex, initial radiotherapy (IniRT), initial systemic treatment (IniST), subsequent radiotherapy (SubRT), and subsequent systemic treatment (SubST) were included, and the genomic characteristics were extracted from the somatic mutation status of each gene. The IniRT was defined as WBRT for treatment strategy when initial diagnosis, and the IniST was defined as systemic chemotherapy treatment. SubRT included (1) WBRT as salvage treatment when the disease was not controlled with initial treatment, and (2) WBRT as consolidation treatment when the disease was under control with initial treatment. SubST included systemic chemotherapy or stem cell transplantation. The somatic mutations of each gene somatic single nucleotide variations (SNVs), insertions, and deletions were identified by WES followed by Sanger sequencing using frozen tissues or from formalin-fixed paraffin-embedded (FFPE) tissues. The detailed description for patient, treatment characteristics, and somatic mutation identification workflow can be found in a previous publication [18]. Overall survival was considered the primary endpoint for the study population. The survival interval was tracked either from the date of diagnosis until the date of death for patients who died within the follow-up period or until the end date of the study for patients who survived. Gene set enrichment analysis for candidate genes was performed to annotate involved gene ontologies and pathways.

### 2.2. Partial Least Squared Path Model (PLS-PM)

PLS-PM can determine the complex relationship between included variables and interest outcomes using structural and measurement models with restricted sample size. Each latent variable was composed of the corresponding manifest variables (clinical or genomic characteristics). The aggregation of manifest variables for specific latent variables is considered as a structural model, and the aggregation of latent variables is considered as a measurement model. In the current study, we used three structural models and one measurement model to demonstrate the impact of included characteristics on overall survival (OS). The measurement model demonstrated the directional relationship between latent variables, including clinical (CLI), somatic mutation (MUT), radiation treatment (TRX), and OS. The structural model for CLI includes age and sex, and the structural model for MUT includes *ROBO1*, *KAT2B*, *SETD1B*, *GNA13*, *APBA1*, and *MYD88*, and the structural model for TRX includes IniRT, IniST, SubRT, and SubST. The factor loadings, cross-loadings, communality, and redundancy of each manifest variable were computed. Concrete variables were selected according to the PLS-PM results and were considered as stratification indicators for OS.

### 2.3. Statistical Analysis

The distribution of clinical and genomic characteristics of the study population was summarized using mean and standard deviation for diagnosis age or summarized using frequency and percentage for other variables. The difference in distribution between PLS-PM-derived subgroups (according to SubRT, *ROBO1*, and *KAT2B* mutation status) was appropriately estimated using Fisher's exact test using the Wilcoxon rank-sum test. In addition, the OS of PLS-PM-derived subgroups was estimated and illustrated using Kaplan-Meier methods and tested using the log-rank test. All analyses were conducted using R 4.0.2 software (R Core Team, 2021), and PLS-PM was performed using the plspm package [19].

## 3. Results

Table 1 summarizes the gene ontologies, including biological processes, molecular functions, and biological pathways involved in candidate genes. This study included genes associated with angiogenesis, tumor microenvironment, cytokines, receptors involving angiogenesis, organelles, and messengers that regulate a myriad of diverse cellular activities.

Table 2 presents the clinical and genomic characteristics of the study population. All characteristics corresponded to the specific latent variables. The mean age of the study population was 67.1 ± 7.7 years, and 8 (44.4%) patients were male. Regarding genomic characteristics, 2 (11.1%) patients were characterized by *ROBO1*, *KAT2B*, *SETD1B*, *GNA13*, and *APBA1* somatic mutations, while six (33.3%) with *MYD88* somatic mutations. In the initial treatment, two (11.1%) patients had received IniRT and 13 (72.2%) patients had received IniST. The somatic mutation profile of the selective gene for each patient is illustrated in Supplementary Figure S1. There are IniRT patients receiving initial WBRT, and there are 12 IniST patients receiving methotrexate-based regimen, one IniST patient receiving nonmethotrexate-based regimen, and three patients without initial treatment. Most of the patients followed the standard treatment guideline which was similar with the current treatment strategy. In subsequent treatment, there are six patients receiving WBRT (four patients as salvage treatment), two patients receiving WBRT combined with rituximab-based regimen, and one patient receiving autologous stem cell transplant as consolidation, and five patients without subsequent treatment. Therefore, six patients who receive subsequent radiotherapy were treated with HD-MTX induction chemotherapy initially.

Figure 1 illustrates the factor loadings and path coefficients of the structural and measurement models using PLS-PM. The ellipse shapes indicate the latent variables (CLI, MUT, TRX, and OS), and the rectangular shapes indicate the manifest variables. The direction of the arrow indicates the direction of the relationship among the variables (either latent or manifest). The blue line and value indicate positive factor loadings between the manifest and latent variables in the outer model. In the CLI structural model, diagnosis age (0.617) and sex (0.856) were both positively related to CLI latent variables. In the TRX structural model, IniRT (0.041) and IniST (0.152) showed a weak positive relationship with TRX latent variables, while SubRT (0.888) and SubST (0.562) also showed a positive relationship with TRX latent variables. In the MUT structural model, *ROBO1* (0.851), *KAT2B* (0.857), *SETD1B* (0.659), *GNA13* (0.715), *APBA1* (0.741), and *MYD88* (0.663) were all positively related to the MUT latent variables. The black line and value indicate positive path coefficients or relations, and the gray line and text indicate negative path coefficients or relations between latent variables in the measurement model. In the measurement model, the CLI latent variable was negatively related to MUT (CLI ➔ MUT, -0.166) latent variables but positively related to TRX (CLI ➔ TRX, 0.666) and OS (CLI ➔ OS, 0.233) latent variables. The MUT latent variable was negatively related to TRX (MUT ➔ TRX, -0.129) and OS (MUT ➔ OS, -0.469) latent variables, while the TRX latent variable was positively related to OS (TRX ➔ OS, 0.096) latent variable.

Table 3 reveals the factor loadings and cross-loadings of each manifest variable in both the structural and measurement models. Higher factor loadings indicate that variability in the manifest variable could better reflect the contribution within the latent variable. A higher communality index and redundancy index indicate a better quality of the measurement model and structural model for each latent variable, respectively. The measurement model results indicated that SubRT, *ROBO1*, and *KAT2B* somatic mutation status had a simultaneously higher redundancy index, communality index (criterion threshold: 0.7), and factor loading value (within the corresponding structural model), which suggests a reasonable quality of the measurement model for OS. Hence, we used SubRT, *ROBO1*, and *KAT2B* somatic mutation status to stratify the study population.

Table 4 summarizes the clinical and genomic characteristics of the study population according to SubRT, *ROBO1*, and *KAT2B* somatic mutation status, regarded as the PLS-PM-derived subgroup. The study population was stratified into no SubRT+mutated, SubRT+nonmutated, and no SubRT+nonmutated subgroups. The no SubRT+mutated subgroup included two patients who have not received SubRT, characterized by *ROBO1* and *KAT2B* somatic mutations. The SubRT+nonmutated subgroup included six patients who received SubRT, but no mutations in *ROBO1* and *KAT2B*. The no SubRT+nonmutated subgroup included ten patients who did not receive SubRT, and no mutations in *ROBO1* and *KAT2B*. Besides the PLS-PM-derived stratification indicators (SubRT, *ROBO1*, and *KATB*), the SubRT+nonmutated subgroup showed a significantly higher proportion in males compared with the no SubRT+mutated and no SubRT+nonmutated subgroups (*P* = 0.027). Other characteristics showed no statistically significant differences between subgroups.  Figure 2 illustrates the Kaplan-Meier curves of the PLS-PM-derived subgroups. Although no statistically significant results were found between subgroups (*P* = 0.780), the no SubRT+nonmutated subgroup showed worse OS compared to the SubRT+nonmutated or SubRT+mutated subgroups in a short-term survival follow-up interval.

## 4. Discussions

The major contribution of this study is that we used a rational statistical approach to analyze a relatively small sample size of lymphoma, PCNSL. This study identified the effects of genes involved in the tumor microenvironment and angiogenesis. This study demonstrated that genes associated with angiogenesis, tumor microenvironment, and chromatin modification were potential indicators of PCNSL survival status and might be affected by the addition of SubRT with induction of HD-MTX chemotherapy.

Consistent with previous reports, angiogenesis plays an important role in PCNSL and leads to vessel neoformation and tumor progression via cytokines, signal transducers, and even chromatin modification [8–10]. Some angiogenesis-related transcription activators, such as STAT3, were expressed at higher levels in tumor PCNSL vessels and cells than in normal brain tissue [17]. Chromatin modification is also involved in the tumorigenesis of PCNSL [20]. The histone lysine methyltransferase, *KMT2D*, has a higher mutation frequency in PCNSL patients than in *de novo* DLBCLs [21, 22]. ROBO1 is mainly expressed in vascular endothelial cells and is involved in angiogenesis through the Slit-Robo signaling pathway [23]. In myeloma study, ROBO1 also regulates the cancer microenvironment by inducing cancer cells to homing, disseminating, and surviving [11]. Blocking Robo activity could inhibit the growth of cancer cell. The lysine acetyltransferase inhibitor was used to modulate the transcriptional activation of KAT2B, to disrupt the tumor angiogenesis acting on both endothelial and tumor cells [12]. Besides, KAT2B also regulated the microenvironment by affecting keratinocyte and stromal cells via nonhistone protein acetylation [13]. Targeting epigenetic changes, including inhibitors of DNA methyltransferase and histone deacetylase (HDAC), are also being investigated and may become a new therapeutic option [24]. Therefore, there is an increasing emphasis on investigating the influence of genes related to angiogenesis and epigenetic modifications.

WBRT has been the mainstay of treatment for PCNSL for decades [25]. WBRT can achieve a high response rate, but remissions are not durable with poor OS [26]. Combination therapy with WBRT and high-dose methotrexate (HD-MTX) improved clinical outcomes, and even HD-MTX replaced WBRT in the treatment of PCNSL [27]. A phase 3 randomized trial, G-PCNSL-SG-1, demonstrated no significant difference in OS when WBRT was omitted from HD-MTX chemotherapy in patients with PCNSL (hazard ratio, 1.06; 95% confidence interval, 0.80-1.40) [7]. However, the disease control may be improved with WBRT (median PFS, 18.3 vs. 11.9 months; *P* = 0.14) [7]. WBRT and autologous stem cell transplantation are considered consolidation therapies [28]. The most serious adverse effect of WBRT is neurotoxicity, including gait disturbances, incontinence, and disabling dementia [29]. The above results were compatible with our findings that patients treated with initial standard HD-MTX chemotherapy and subsequent WBRT demonstrated a trend of better outcomes in our analysis.

PLS-PM has less stringent assumptions on sample size distribution, which could provide a nonparametric approach to infer model-based relationships and interaction effects between observed factors and outcomes using a small sample size [30–32]. In addition, PLS-PM can estimate the complex relationship between manifest and latent variables via a data-driven exploration procedure based on the causal interpretability assumption [33]. In this study, PLS-PM successfully used a limited sample size to derive a survival-associated subgroup in PCNSL based on clinical characteristics, treatment modalities, and genomic alterations.

Nevertheless, there are some limitations to this study. First, the clinical characteristics of the patients were limited to the data set. The prognostic index of the International Extranodal Lymphoma Study Group (IELSG) was not evaluated in our study. The prognostic index of IELSG, including performance status, serum LDH level, cerebrospinal fluid protein, and the involvement of deep structure, was a prognostic tool for distinguishing risk groups in immunocompetent patients with PCNSL [34]. Second, the retrospective nature of this study limited the inclusion of factors associated with survival in patients with PCNSL. Third, although the influence of survival time was ignored in PLS-PM, Kaplan-Meier methods were used to further confirm the survival difference between PLS-PM-derived subgroups. Despite these limitations, this study contributes findings, including those from the investigation of the impact of the tumor microenvironment and angiogenesis-associated genomic alterations and treatment modalities on the OS of patients with PCNSL.

## 5. Conclusions

This is the first study using PLS-PM to investigate the influence of genomic alterations and treatment modalities on the survival of PCNSL. The study findings indicate that patients with no mutations of *ROBO1* and *KAT2B*, the SubRT subgroup showed favorable survival outcomes compared with the no SubRT subgroup in short-term follow-up. Since all SubRT patients receiving high-dose methotrexate induction chemotherapy in initial treatment, hence, initial standard HD-MTX chemotherapy with subsequent WBRT could potentially improve the survival outcome in PCNSL patients who have no ROBO1 and KAT2B somatic mutations in short-term follow-up. Therefore, the overall findings suggest that angiogenesis and the tumor microenvironment play important roles in the prognosis of PCNSL. However, it is necessary to use a comprehensive pathophysiological approach to elucidate the complex relationship between prognostic gene alterations and treatment modalities to encourage precise predictions of PCNSL.

## Figures and Tables

**Figure 1:** The partial least squared path model demonstrates the impact of clinical (CLI), somatic mutation (MUT), and radiation treatment (TRX) on overall survival (OS). CLI, MUT, TRX, and OS were defined as latent variables (ellipse), and the corresponding manifest variables (rectangle) were connected using arrow lines. The direction of arrow indicates the direction of the relation among the variables (either latent or manifest). Black line and value indicate positive path coefficients or relation, whereas gray line and text indicate negative path coefficients or relation between latent variables in the measurement model. Blue line and value indicate positive factor loadings between manifest and latent variables in the structural model.

**Figure 2:** Kaplan-Meier plot according to SubRT, *ROBO1*, and *KAT2B* somatic mutation status.

**Table 1:** Biological process, molecular functions, and KEGG pathways of candidate genes.

Category	Genes in pathway	*P* value	FDR	% in pathway	Genes
Biological process					
GO:0002042~cell migration during sprouting angiogenesis	4	0.003	0.008	25.0	ROBO1
GO:0016568~chromatin modification	104	0.004	0.008	1.9	KAT2B; SETD1B
GO:0001569~patterning of blood vessels	8	0.007	0.008	12.5	GNA13
GO:0035264~multicellular organism growth	8	0.007	0.008	12.5	APBA1
GO:0043542~endothelial cell migration	8	0.007	0.008	12.5	ROBO1
Molecular function					
GO:0031701~angiotensin receptor binding	5	0.004	0.007	20.0	GNA13
GO:0031702~type 1 angiotensin receptor binding	5	0.004	0.007	20.0	GNA13
GO:0005546~phosphatidylinositol-4,5-bisphosphate binding	7	0.006	0.007	14.3	APBA1
Biological pathways^1^					
IL-1 signaling	91	0.003	0.007	2.2	GNA13; MYD88

^1^Biological pathways were annotated according to the Kyoto Encyclopedia of Genes and Genomes (KEGG) library. FDR: false discovery rate.

**Table 2:** Clinical and genomic characteristics of study population.

Latent variables	Manifest variables	Description	Overall (*n* = 18)
CLI	AGE (mean ± SD)	Diagnosis age	67.1 ± 7.7
CLI	SEX (male)	Sex	8 (44.4%)
MUT	ROBO1	Candidate gene	2 (11.1%)
MUT	KAT2B	Candidate gene	2 (11.1%)
MUT	SETD1B	Candidate gene	2 (11.1%)
MUT	GNA13	Candidate gene	2 (11.1%)
MUT	APBA1	Candidate gene	2 (11.1%)
MUT	MYD88	Candidate gene	6 (33.3%)
TRX	IniRT	Initial radiotherapy	2 (11.1%)
TRX	IniST	Initial systemic treatment	13 (72.2%)
TRX	SubRT	Subsequent radiotherapy	6 (33.3%)
TRX	SubST	Subsequent systemic treatment	3 (16.7%)

**Table 3:** Factor loadings and cross-loadings of each manifest variable in measurement model.

Manifest variables	Latent variables	CLI	MUT	TRX	OS	Communality	Redundancy
AGE	CLI	0.617	-0.232	0.240	0.242	0.38	<0.01
SEX	CLI	0.856	-0.057	0.710	0.316	0.73	<0.01
ROBO1	MUT	-0.008	0.851	-0.270	-0.438	0.72	0.02
KAT2B	MUT	-0.008	0.851	-0.270	-0.438	0.72	0.02
APBA1	MUT	-0.218	0.741	-0.164	-0.438	0.55	0.02
GNA13	MUT	-0.216	0.715	-0.020	-0.438	0.51	0.01
MYD88	MUT	-0.205	0.663	-0.187	-0.125	0.44	0.01
SETD1B	MUT	-0.107	0.659	-0.164	-0.438	0.43	0.01
IniRT	TRX	0.249	0.151	0.041	0.125	<0.01	<0.01
IniST	TRX	-0.210	-0.134	0.152	-0.219	0.02	0.01
SubRT	TRX	0.597	-0.252	0.888	0.250	0.79	0.39
SubST	TRX	0.093	-0.184	0.562	0.158	0.32	0.15
OS	OS	0.377	-0.531	0.368	1.000	—	—

**Table 4:** Clinical and genomic characteristics of study population according to subsequent SubRT, *ROBO1*, and *KAT2B* somatic mutation status.

Characteristic	No SubRT+mutated (*n* = 2)	SubRT +nonmutated (*n* = 6)	No SubRT+nonmutated (*n* = 10)	*P* value
AGE (mean ± SD)	65.5 ± 16.3	70.3 ± 6.6	65.5 ± 6.9	0.500
SEX (male)	1 (50.0%)	5 (83.3%)	2 (20.0%)	0.027
ROBO1	2 (100.0%)	0 (0.0%)	0 (0.0%)	0.007
KAT2B	2 (100.0%)	0 (0.0%)	0 (0.0%)	0.007
APBA1	1 (50.0%)	0 (0.0%)	1 (10.0%)	0.314
GNA13	1 (50.0%)	1 (16.7%)	0 (0.0%)	0.085
MYD88	2 (100.0%)	1 (16.7%)	3 (30.0%)	0.193
SETD1B	1 (50.0%)	0 (0.0%)	1 (10.0%)	0.314
IniRT	0 (0.0%)	0 (0.0%)	2 (20.0%)	0.608
IniST	1 (50.0%)	6 (100.0%)	6 (60.0%)	0.212
SubRT	0 (0.0%)	6 (100.0%)	0 (0.0%)	<0.001
SubST	0 (0.0%)	2 (33.3%)	1 (10.0%)	0.669
OS	1 (50.0%)	6 (100.0%)	9 (90.0%)	0.314

*P* value is estimated using the Wilcoxon rank-sum test or Fisher's exact test.

## Data Availability

The data that support the findings of this study are openly available in cBioPortal at https://www.cbioportal.org/study/summary?id=pcnsl_mayo_2015.

## Supplementary Materials

Supplementary Materials Supplementary Figure S1: the somatic mutation profile of the selective gene for each patient.
